The article "Diagnostic Value of SonoVue Contrast-Enhanced Ultrasonography in Nipple Discharge Based on Artificial Intelligence" was retracted in 2023. Reasons: signs of a paper mill; compromised peer review; unreliable results or conclusions.

# Diagnostic Value of SonoVue Contrast-Enhanced Ultrasonography in Nipple Discharge Based on Artificial Intelligence

**DOI:** 10.1155/2021/2961697

**Published:** 2021-12-16

**Authors:** Ling Guo

**Affiliations:** Pingxiang People's Hospital, Pingxiang 337000, China

## Abstract

This paper aims to explore the application value of SonoVue contrast-enhanced ultrasonography based on deep unsupervised learning (DNS) in the diagnosis of nipple discharge. In this paper, a new model (ODNS) is proposed based on the unsupervised learning model and stack self-coding network. The ultrasonic images of 1,725 patients with breast lesions in the shared database are used as the test data of the model. The differences in accuracy (Acc), recall (RE), sensitivity (Sen), and running time between the two models before and after optimization and other algorithms are compared. A total of 48 female patients with nipple discharge are enrolled. The differences in SE, specificity (SP), positive predictive value (PPV), and negative predictive value (NPV) of conventional ultrasound and contrast-enhanced ultrasonography are analyzed based on pathological examination results. The results showed that when the number of network layers is 5, the classification accuracies of DNS and ODNS model data reached the highest values, which were 91.45% and 98.64%, respectively.

## 1. Introduction

Nipple discharge is one of the three common symptoms of female breast diseases. About 3%–10% of patients complained of nipple discharge in the outpatient department of the hospital [1]. Therefore, the number of patients undergoing surgical treatment is only second to that of patients with breast masses [2]. The nipple discharge includes physiological and pathological nipple discharge. Pathological nipple discharge is often manifested as spontaneous and serous discharge, mainly caused by trauma, inflammation, intraductal papilloma, ductal dilatation, and papillomatosis. Intraductal papilloma is a common pathological type, accounting for about 57% of pathological nipple discharge [3]. At present, breast molybdenum target, breast color Doppler ultrasound, galactography, and cytology are often used for the diagnosis of nipple discharge. Since patients with nipple discharge are often not accompanied by breast masses or masses are too small, the results of molybdenum target and color Doppler ultrasound are often negative [4]. The exfoliated cells of nipple discharge are commonly used in clinical examination of breast diseases, but its sensitivity is low [5]. The operation of galactography is simple and completely noninvasive and can directly observe the morphology of mammary duct. However, the results are susceptible to factors such as extrusion and breast size, and the false positive rate is as high as 20%–30% [6]. Ultrasound examination is widely used in the diagnosis of various diseases due to its real time, being nonradioactive, and low price. High-frequency ultrasound can display the morphology and relationship of dilated breast duct, duct, and surrounding glands, and the sensitivity of pathological nipple discharge diagnosis can reach 97% [7].

With the continuous development of artificial intelligence technology, deep learning is widely used in image processing, speech recognition, and big data mining. Deep learning is a process of running a series of supervised or unsupervised learning algorithms [8]. Traditional data analysis labels data in the way of supervised learning and then trains its parameters. However, labeling all data for big data makes the task very complicated, and its training effect is limited [9]. Unsupervised learning algorithm has excellent feature learning ability, which is conducive to data classification [10]. Some studies pointed out that, in the process of unsupervised initialization, the introduction of greedy layer-by-layer unsupervised training method can improve the generalization performance of big data [11]. However, unsupervised deep learning is limited by computer hardware in the process of big data training, resulting in slow convergence [12].

In this paper, based on the superior generalization ability and excellent feature learning method of unsupervised learning method, it is optimized to increase its classification efficiency, and it is applied to the diagnosis of patients with nipple discharge. 48 female patients with nipple discharge were selected as the research objects to explore the application value of SonoVue galactography based on the optimized unsupervised learning model in the diagnosis of nipple discharge, so as to provide reference for the diagnosis and treatment of nipple discharge.

## 2. Materials and Methods

### 2.1. Unsupervised Deep Learning Model Establishment

For the same size feature set, deep network has more parameters than shallow network, which leads to underfitting and overfitting of deep network learning [13]. The single neural source of unsupervised deep learning mainly includes synapse, adder, and activation function [14]. Assuming that the corresponding linear regression model is established when the activation function is linear transformation *α*(*x*)=*x*, the regression vector composed of the input data can be expressed as follows:

(1) $$\begin{array}{c} X={\left[x_{1},x_{2},\ldots ,x_{n}\right]}^{A}, \end{array}$$

where *A* is the transpose of the matrix and *n* is the number of features. The output *b* of a single neuron can be expressed as equation (2), where *β* is bias and *ω* is synaptic weight.

(2) $$\begin{array}{c} b=\sum_{i=1}^{n}\omega_{i}x_{i}+\beta . \end{array}$$

Considering a series of data [*x*^(*i*)^, *y*^(*i*)^],  (*i*=1,2,…, *m*), its input data *x* ∈ *R*^*N*_1_^, and expected output data *y* ∈ *R*^*N*_2_^, the performance metrics of the data can be expressed as follows:

(3) $$\begin{array}{c} E=\frac{1}{2m}\sum_{i}{\left[y^{\left(i\right)}-b^{\left(i\right)}\right]}^{2}=\frac{1}{2}B\left[{\left\|Y-C\right\|}^{2}\right], \end{array}$$

where *m* is the number of training data pairs, *Y* is the expected output data vector, *C* is the output vector of training data, and *E* is the loss function.

Suppose that the number of neurons is *L*; then the *j* neurons can be expressed as follows:

(4) $$\begin{array}{c} d_{j}^{l}=\chi \left(\sum_{k}\omega_{jk}^{l}d_{k}^{l-1}+c_{j}^{l}\right). \end{array}$$

*ω*_*jk*_^*l*^ represents the weight value of the *k* neurons in the *l* − 1 layer to the *j* neurons in the *l* layer, and *c*_*j*_^*l*^ represents bias *χ* of the *j* neurons in the *l* layer as the activation function; *χ*(*z*)=(1/1+*e*^−*z*^).

Assuming that the error of the *j* neuron in the *l* layer is *δ*_*j*_^*l*^, the calculation method is as follows:

(5) $$\begin{array}{c} \delta_{j}^{l}=\frac{\partial D}{\partial z_{j}^{l}}. \end{array}$$

Assuming that the error of the *l* layer neuron is *δ*^*l*^, the calculation method is as follows:

(6) $$\begin{array}{c} \delta^{l}=\left[{\left(\omega^{l+1}\right)}^{T}\delta^{l+1}\right]⊙\chi {}^{\prime }\left(z^{l}\right). \end{array}$$

⊙ is the Hadamard product, *χ*′(*z*^*l*^) is the output vector of the nonlinear transformation of the activation function, and the *δ*^*l*^ matrix can be expressed as follows:

(7) $$\begin{array}{c} \delta^{l}=\text{Diag}\left[\chi {}^{\prime }\left(z^{l}\right)\right]\left(\omega^{l+1}\right)\delta^{l+1}. \end{array}$$

Diag[*χ*′(*z*^*l*^)] is the principal diagonal matrix composed of *χ*′(*z*^*l*^).

The *χ*′(*z*^*l*^) calculation method can be obtained according to the calculation method of activation function.

(8) $$\begin{array}{c} \chi {}^{\prime }\left(z^{l}\right)=\frac{1}{e^{-z}{\left(1+e^{-z}\right)}^{2}}. \end{array}$$

The gradient descent method always finds the local minimum closest to the initial point and then obtains the global optimal solution [15]. Assuming that the random initialization *ω* of the gradient descent method obeys the standard normal distribution, *ω*_*jk*_^*l*+1^ ≤ 1.

(9) $$\begin{array}{c} \delta^{l}=\chi {}^{\prime }\left(z_{j}^{l}\right)\omega_{jk}^{l+1}\chi {}^{\prime }\left(z_{k}^{l+1}\right)\omega_{jk}^{l+2}\cdots \chi {}^{\prime }\left(z_{k}^{L}\right)\frac{\partial D}{\partial {\text{z}}^{L}}\leq {\left(\frac{1}{4}\right)}^{N}\frac{\partial D}{\partial {\text{z}}^{L}}. \end{array}$$

In the equation, *N* is the number of layers from *l* layer to *L* layer.

The data samples are input into the input layer of the unsupervised learning model, and the hidden layer is processed by the input layer. Then, the global optimal solution is calculated by the gradient descent method, and it is input to output layer, which is processed by the output layer to output the results. The process of unsupervised deep learning model algorithm is shown in Figure 1.

### 2.2. Unsupervised Deep Learning Model Optimization

In the supervised deep learning, the learning of parameters depends on the label data, which makes it difficult to obtain sufficient label samples, increases the cost of manpower and financial resources, and significantly reduces the generalization ability of data [16]. The initial value sensitivity of unsupervised learning data acquisition process makes the gradient descent method fall into the local extremum problem and makes the parameters difficult to train [17]. In the process of network feature learning, the self-coding learning method is used to process the data.

Assuming that *f*[*α*(*x*)] ≈ *x*, the input data *x* is encoded to approximate input value $\tilde{x}$ in the decoding process, *α*(*x*) is encoding, *f*(*x*) is decoding, and the output data $\tilde{x}$ can be expressed as follows:

(10) $$\begin{array}{c} \tilde{x}=Hy, \end{array}$$

where *H* is the matrix composed of hidden layer neurons output *h*_*i*_, *H*=[*h*_1_, *h*_2_,…, *h*_*L*_], and *y* is the coefficient vector.

When the number of neurons in the hidden layer is large, the feature data of the self-coded network can be expressed as the following equation, where *h*_*k*_ is the image edge information matrix element obtained by sparse self-encoder learning, $\tilde{h_{i}^{l}}$ is the input data, and *h*_*k*_^*l*+1^ is the feature data.

(11) $$\begin{array}{c} \tilde{h_{i}^{l}}=\sum_{k=1}^{H}y_{ik}^{l}h_{k}^{l+1}. \end{array}$$

The data reconstructed after encoding and decoding by the self-encoder can be expressed as follows:

(12) $$\begin{array}{c} \tilde{h_{i}^{l}}=\sum_{k=1}^{H}y_{ik}^{l}\eta \left(\sum_{i=1}^{D}\omega_{ik}^{l+1}h_{i}^{l}\right), \end{array}$$

where *h*^*l*^ is input data and *D* is feature dimension for input data.

Sparse self-coding algorithm tries to find the reconstruction close to the input to be mathematically expressed as follows:

(13) $$\begin{array}{c} {\left\|\tilde{h}-h\right\|}^{2}⟶0. \end{array}$$

When the number of training samples is *m*, the loss function *E* can be expressed as follows:

(14) $$\begin{array}{c} E=\frac{1}{2m}\sum_{i=1}^{m}{\left\|\tilde{h}\left[h^{\left(i\right)},\omega ,y\right]-h^{\left(i\right)}\right\|}^{2}⟶0. \end{array}$$

In order to obtain the optimal solution of the above equation *ω* and *y*, the expression used to solve the optimal problem is shown below:

(15) $$\begin{array}{c} \min\frac{1}{2m}\sum_{i=1}^{m}{\left\|\tilde{h}\left[h^{\left(i\right)},\omega ,y\right]-h^{\left(i\right)}\right\|}^{2}+\frac{\kappa }{2m}\sum_{i=1}^{m}{\left\|y\right\|}^{2}. \end{array}$$

The equation (*κ*/2*m*)∑_*i*=1_^*m*^‖*y*‖ is a sparse penalty function and *ω* is a weight coefficient.

Deep network learning is composed of multilayer networks, so it is necessary to stack the self-coded network of single hidden layer [18]. The stacked self-coded network is composed of multilayer autoencoders. The output of the front layer autoencoder can be used as the input of the back layer autoencoder. The encoding of the stacked self-coded network can be expressed as follows:

(16) $$\begin{array}{c} h^{l+1}=\eta \left(\omega^{l+1}h^{l}+b^{l+1}\right), \end{array}$$

where *l*=1,2,…, *L*; then the optimization problem of the stacked self-coded network is expressed as follows:

(17) $$\begin{array}{c} \min\frac{1}{2m}\sum_{i=1}^{m}{\left\|\tilde{h}\left(h^{l}\right)-h^{l}\right\|}^{2}+\frac{\kappa }{2m}\sum_{i=1}^{m}{\left\|y^{l}\right\|}^{2}. \end{array}$$

Deep network parameter learning from global optimization is a common strategy for weight coefficient optimization. In this study, the weights of neurons in all network layers were optimized by the back-propagation of errors. In order to calculate the gradient of all layers in each iteration, a Softmax classifier can be added to the L-1 layer of the deep network to adjust the weight value, and the optimized model is named optimized unsupervised deep learning.

The optimized unsupervised deep learning model preprocesses the input image by the encoder in the self-coding model and then processes the input layer, hidden layer, and output layer of the self-coding model, processes the image by the decoder, and finally outputs the medical image of feature classification. Optimized unsupervised deep learning image processing is shown in Figure 2.

For large data sets, the “big data + complex model” mode can effectively improve learning efficiency [19]. Therefore, this study introduces the Mini-Batch gradient descent algorithm to optimize the unsupervised learning model in the processing of large data sets. For each sample *k*=1,2,…, *K*, the iterative equation after the Mini-Batch gradient descent algorithm is as follows:

(18) $$\begin{array}{c} \tilde{\omega_{ij}^{i}}=\omega_{ij}^{i}-\frac{\eta }{b}\sum_{k=1}^{1+b}\left[y^{\left(k\right)}-h^{L}\left[x^{\left(k\right)},\omega \right]\right]\frac{\partial h^{L}}{\partial \omega_{ij}^{L}}, \end{array}$$

where *b* is the size of each selected small batch sample data set.

### 2.3. Model Test Data and Results Evaluation

The medical images of the model test set are mainly ultrasound images, which were all from the shared database of the imaging department of the hospital. The collected data were from 1,725 patients with breast lesions. The images included in this study met the following criteria: (1) The ultrasound images of all patients were breast scanning images. (2) Image quality is clear. (3) Data on patients included in the study were complete. To protect patient privacy, the database anonymously processes all patients' personal information using data encryption and all patients or their families signed informed consent. The research process is approved by XX hospital ethics committee. The computer hardware is configured as Intel dual-core Xeon CPU and the main frequency is 3.4 GHz, with 8.0 GB memory, 1 TB hard disk, and 512 MB display card. The experiments were implemented in Matlab7.0 software environment.

In this study, the accuracy (Acc), recall (RE), sensitivity (Sen), and runtime analysis model were used to classify the test set. The calculation methods of Acc, RE, and Sen were as follows:

(19) $$\begin{array}{c} \text{Acc}=\frac{\text{TP}+\text{TN}}{\text{TP}+\text{FN}},\\ \text{RE}=\frac{\text{TP}}{\text{TP}+\text{FN}},\\ \text{Sen}=\frac{\text{TP}}{\text{TP}+\text{FN}}. \end{array}$$

TP represents the number of correct classification results. FN represents the number of missed classifications. TN represents the number of misclassifications. FP represents the number of wrong classification results.

### 2.4. Research Objects and Grouping

From January 2020 to December 2020, 48 female patients who received surgical treatment in Pingxiang People's Hospital due to nipple discharge were enrolled as the research objects. The age of patients ranged from 10 to 63 years, with an average age of 43.75 ± 6.02 years. The inclusion criteria of this study were as follows: (1) patients diagnosed as pathological nipple discharge, (2) patients with ipsilateral breast and no history of surgical treatment, and (3) patients who underwent SonoVue galactography. Exclusion criteria were as follows: (1) patients with physiological nipple discharge; (2) patients without breast lumps; (3) patients with heart, lung, brain, or other important organ dysfunctions, and (4) patients in pregnancy or lactation. The study process is approved by the Pingxiang People's Hospital ethics committee, and the subjects included in the study signed informed consent.

### 2.5. Method and Result Analysis of Galactography

The patients were examined by conventional ultrasound with Philips iU22 color Doppler ultrasound diagnostic instrument before galactography. The patients were taken in supine position and the nipple was taken as the center to observe the dilated duct, hypoechoic nodules, and bilateral axillary lymph nodes. 3 mL contrast agent was taken to detect the patency of lacrimal irrigation needle, the nipple surface debris and condensate overflow were removed, and SonoVue contrast agent was injected slowly. When the patient complained of mild swelling and pain, the injection was stopped, and the mechanical index was adjusted to a lower state. Contrast-enhanced ultrasound is performed on the lesion area to observe the state of the breast duct and its interruption.

The pathological examination results were used as the diagnostic criteria, and the results of SonoVue ultrasound and conventional ultrasound were compared and analyzed to evaluate the sensitivity and specificity, positive predictive value, and negative predictive value of SonoVue ultrasound and conventional ultrasound. The calculation methods of sensitivity, specificity, positive predictive value, and negative predictive value are as follows:

(20) $$\begin{array}{c} \text{SE}=\frac{\text{TP}}{\text{TP}+\text{FN}}\times 100\%,\\ \text{SP}=\frac{\text{TN}}{\text{TN}+\text{FP}}\times 100\%,\\ \text{PPV}=\frac{\text{TP}}{\text{TP}+\text{FP}}\times 100\%,\\ \text{NPV}=\frac{\text{TN}}{\text{FN}+\text{TN}}\times 100\%. \end{array}$$

TP represents the number of true positive diagnosis results. FN represents the number of false negative diagnosis results. TN represents the number of true negative diagnosis results. FP represents the number of false positive results. FN represents the number of false negative diagnosis results.

### 2.6. Statistical Methods

The experimental data were processed by SPSS 20.0 statistical software. The measurement data were subjected to normal distribution test, expressed as mean ± standard deviation ($\bar{x}$ ± *s*), and *t*-test was used for comparison between groups. The pathological type results of patients with nonnormal distribution were tested by nonparametric test, and the enumeration data were expressed as percentage (%), and *χ*^2^ test was used. *P* < 0.05 indicated that the difference was statistically significant.

## 3. Results

### 3.1. Analysis of Test Results of Unsupervised Deep Learning Model

The accuracy and running time of test set classification under different network layers are analyzed, as shown in Figure 3. When the number of network layers is in the range of 1–5, with the increase of network layers, the accuracy of test set data classification showed a significant upward trend. When the number of network layers was 5, the accuracy of data classification reached 91.45%. When the number of network layers was greater than 6, with the increase of network layers, the accuracy of test set data classification showed a significant downward trend. When the number of network layers was 10, the accuracy was 5.50%. With the increase of network layers, the running time of test set data classification was significantly increased.

The correlation between the weight coefficient and the number of iterations under different network layers of the optimized unsupervised deep learning model is analyzed, as shown in Figure 4. With the increase of the number of iterations, the weight coefficient under different network layers (N1–N9) showed a significant downward trend. Under the same iteration number, with the increase of the number of network layers, the weight coefficient showed a significant increase trend. When the number of iterations was 1 and the number of network layers was 10, the weight coefficient reached the maximum of 0.98.

### 3.2. Test Results Analysis of Optimized Unsupervised Deep Learning Model

The accuracy and recall rate of test set classification under different network layers of the optimized model are analyzed, as shown in Figure 5. With the increase of network layers, the accuracy of test set data classification increased first and then decreased. When the number of network layers was 5, the accuracy of data classification reached the maximum of 98.64%. When the number of network layers was greater than 6, the accuracy of test set data classification decreased with the increase of network layers. When the number of network layers was 10, the accuracy reached the lowest value of 83.67%. There is no significant difference in the accuracy of data set classification under different network layers.

The loss curve before and after the optimization of the unsupervised deep learning model is analyzed, as shown in Figure 6. When the training time was 30 min, the accuracy of the model was 98.64% at 15 min, while the accuracy of the unoptimized model was only 70.69% at 15 min, and the highest accuracy of the model was 92.75% at 30 min.

The classification accuracy and sensitivity of the optimized unsupervised deep learning model, perceptron model, deep belief network (DBN), and random Boolean neural network in this study were compared, as shown in Figure 7. The maximum Acc value of unsupervised deep learning model is 96.67 ± 0.45%, which is significantly higher than 91.52 ± 0.57%, 92.08 ± 0.33%, and 94.35 ± 0.64% of perceptron model, DBN, and random Boolean neural network, respectively. The Spe value of unsupervised deep learning model is 87.24 ± 1.15%, which is significantly higher than those of perceptron model, DBN, and random Boolean neural network: 72.14 ± 1.22%, 70.09 ± 1.34%, and 81.32 ± 0.97%, respectively.

The recall and precision curves of different algorithms were analyzed, as shown in Figure 8. Different algorithms achieved high accuracy and recall levels for the classification results of the training set, while the Acc and RE levels of the optimized unsupervised deep learning model were significantly better than those of other algorithms.

### 3.3. SonoVue Galactography Image Analysis of Nipple Discharge Patients

Galactography images of normal breast duct showed that the outer edge of the breast branch was gradually thinning, the contrast agent filling in the breast duct was uniform and continuous, the branch was natural, and there were no signs of defect, interruption, or expansion in the duct, as shown in Figure 9(a). The contrast-enhanced images of patients with pathological nipple discharge showed catheter dilation, as shown in Figure 9(b). The main duct or secondary and tertiary ducts were significantly interrupted, as shown in Figure 9(c), and hypoechoic nodules were visible, as shown in Figure 9(d). At the same time, patients were accompanied by single or multiple filling defects, as shown in Figure 9(e). The contrast agent in the hypoechoic area of the capsule is filled, and the filling defect area is visible on the wall of the capsule, as shown in Figure 9(f).

### 3.4. Comparison of Diagnostic Results between SonoVue Galactography and Conventional Ultrasound

Among the 48 patients included in this study, 26 (54.17%) hypoechoic nodules were detected by conventional ultrasound, as shown in Figure 10. Among them, 10 (20.83%) hypoechoic nodules were located in the duct, 9 (18.75%) hypoechoic nodules were located outside the duct, and 7 (14.58%) were undetermined. There were 7 cystic-solid nodules (14.58%), of which 4 (8.33%) were located in the duct, and the remaining 3 (6.25%) were undetermined. The results of galactography showed that 14 (29.17%) of the 26 hypoechoic nodules were intraductal lesions, and 12 (25.00%) were extrahepatic lesions. Among the 7 cystic-solid nodules, 5 (10.42%) were intraductal lesions and 2 (4.17%) were extraductal lesions. The proportion of patients with hypoechoic nodules in the results of SonoVue galactography is significantly higher than that in the results of conventional ultrasound (*P* < 0.05).

### 3.5. Clinical Features of Patients

Statistical analysis is performed on the basic clinical features of all patients, as shown in Figure 11. Among all patients, 32 patients (66.67%) were above 50 years of age, 29 patients (60.42%) had left overflow, 45 patients (93.75%) had fertility history, 42 patients (87.5%) had lactation history, and only 8 patients (16.67%) had breast disease history. Among all the patients, 26 patients (54.17%) had serous nipple discharge, 12 patients (25%) had bloody nipple discharge, 8 patients (16.67%) had milky white nipple discharge, and 2 patients (4.17%) had clear water-like nipple discharge.

### 3.6. Comparison of Different Imaging Diagnosis of Nipple Discharge Results

The pathological diagnosis results were used as the gold standard to compare the results of conventional ultrasound diagnosis and SonoVue galactography, as shown in Figure 12. The SE value, SP value, PPV value, and NPV value of conventional ultrasound in the diagnosis of nipple discharge were 77.08%, 58.33%, 83.33%, and 31.25%, respectively. The SE value, SP value, PPV value, and NPV value in the diagnosis of nipple discharge by SonoVue galactography were 100%, 68.75%, 91.67%, and 100%, respectively. The SE value, SP value, PPV value, and NPV value in the diagnosis of nipple discharge by SonoVue galactography were higher than those by conventional ultrasound. The SE value in the diagnosis of nipple discharge by SonoVue galactography is significantly higher than that by conventional ultrasound (*P* < 0.05), and the NPV value in the diagnosis of nipple discharge by SonoVue galactography is higher than that by conventional ultrasound (*P* < 0.01).

## 4. Discussion

In this study, the optimized unsupervised deep learning model is optimized by unsupervised learning method, and the ultrasonic image is used as the test set to analyze it. The results showed that, with the increase of the number of network layers, the accuracy of data classification in the test set is significantly increased. When the number of network layers was 5, the accuracy of data classification reached 98.45%, and when the number of network layers was 10, the accuracy was 5.50%. This suggested that the unsupervised deep learning model has good classification effect. The current research results show that unsupervised deep learning has more powerful feature learning ability than neural network algorithm [20]. The research results of this study are different from the current research results, and the reason is due to the gradient instability. In the process of data processing, supervised deep learning algorithm uses gradient descent algorithm to increase its sensitivity to the initial value [21] and finally makes the training of unsupervised deep learning model parameters more difficult [22]. Unsupervised deep learning model results showed that, with the increase of the number of iterations, the weight coefficient under different network layers represented a significant downward trend. When the number of iterations was 1 and the number of network layers was 10, the weight coefficient reached the maximum of 0.98. This indicated that, in the process of infinitely approaching the convergence of the algorithm, the weight coefficient of the model is getting smaller and smaller, which makes it fall into a pause in the process of training the shallow network of parameters, resulting in the results' bias [23]. Moreover, the asymmetric learning of network parameters at different levels led to a significant increase in running time [24]. Based on the problems of unsupervised deep learning model, sparse self-encoder, stacked self-coding network, and back-propagation algorithm were introduced to optimize it and establish the optimized unsupervised deep learning model. The results showed that, with the increase of network layers number, the accuracy of optimized unsupervised deep learning test set data classification increased first and then decreased. When the network layers number was 5, the accuracy of data classification reached the maximum of 98.64%. When the network layers number was greater than 6, with the increase of network layers number, the accuracy of test set data classification decreased. When the network layers number was 10, the accuracy reached the lowest value of 83.67%. Under different network layers, the accuracy of data set classification had no significant difference. The results revealed that the feature learning ability of optimized unsupervised deep learning is obviously improved. The reason is that the introduction of sparse self-encoder in the optimization process can reduce the superposition of elements [25], and the improved weight coefficient is obtained. In addition, the introduction of stacked self-encoder network improved the feature analysis of the data and obtained the prior information of the data. Finally, the feature learning ability of optimized unsupervised deep learning is improved.

Ultrasonic examination is a commonly used examination method for breast diseases, which has the advantages of no radiation, noninvasiveness, and display of ductal ectasia, but it has limitations in the diagnosis of multiple ductal ectasia [26]. SonoVue galactography is used in clinical nonvascular ultrasound imaging examination [27], and the specificity and sensitivity of transvaginal 3D contrast-enhanced ultrasound reached the standard of laparoscopic tubal fluid staining [28]. In this study, contrast-enhanced ultrasound examination is performed on the basis of ultrasound. The results showed that 26 patients (54.17%) had serous nipple discharge, 12 patients (25%) had bloody overflow, 8 patients (16.67%) had milk-white overflow, and 2 patients (4.17%) had clear water-like overflow. This indicated that most patients with nipple discharge had serous nipple discharge, which is consistent with the results of Jung et al. (2019) [29]. The results in this study showed that the SE value in the diagnosis of nipple discharge by SonoVue galactography is significantly higher than that by conventional ultrasound (*P* < 0.05), and the NPV value in the diagnosis of nipple discharge by SonoVue galactography is higher than that by conventional ultrasound (*P* < 0.01). Compared with conventional ultrasound, the accuracy of nipple discharge is significantly increased.

## 5. Conclusion

In this study, the unsupervised learning model is preliminarily established, and the optimized unsupervised deep learning model is optimized based on the problems existing in the training process, which is applied to the diagnosis of patients with nipple discharge by SonoVue galactography. The results showed that the data processing performance of optimized unsupervised deep learning model is significantly improved, and the sensitivity and negative predictive value of SonoVue galactography in nipple discharge were higher. However, there are still some shortcomings in this study. The patients included in this study are better, and the benign and malignant degrees of intraductal space-occupying lesions in patients are not identified based on the results of SonoVue galactography. In the future, the number of cases will be increased. Based on SonoVue galactography, combined with nipple discharge biomarkers, the benign and malignant diseases of nipple discharge are further identified to provide a more powerful basis for accurate diagnosis of nipple discharge. In conclusion, this study establishes an efficient unsupervised learning model for data classification, and SonoVue galactography has potential application value in nipple discharge, which provides a noninvasive safety inspection method for clinical diagnosis and treatment of nipple discharge.

## Figures and Tables

**Figure 1:** Unsupervised deep learning model process.

**Figure 2:** Optimized unsupervised deep learning model image processing flow.

**Figure 3:** Analysis of model accuracy and running time under different network layers.

**Figure 4:** Trend chart of weight coefficient under different iterations.

**Figure 5:** Analysis of the accuracy and recall rate of the optimized model under different network layers.

**Figure 6:** Loss curves of different algorithms.

**Figure 7:** Comparison of accuracy and specificity of different algorithms.

**Figure 8:** Recall rate and precision curve of different algorithms.

**Figure 9:** SonoVue galactography images of nipple discharge patients. (a) Galactography of normal breast duct. (b) A 31-year-old patient with right breast single-hole bloody spill. (c) A 40-year-old patient with left breast single-hole serous effusion. (d) A 56-year-old patient with left breast single-hole serous effusion. (e) A 38-year-old patient with right breast single-hole hemorrhagic nipple discharge. (f) A 42-year-old patient with left breast single-hole milky white nipple discharge.

**Figure 10:** Analysis of location determination results of breast nodules in different examination methods (^*∗*^represents a statistically significant difference compared with conventional ultrasound, *P* < 0.05).

**Figure 11:** Statistical graph of basic clinical features. (a) Statistical graph of patients' age, overflow side, childbearing history, and breastfeeding history. (b) Statistical graph of the history of breast disease and the proportion of overflow features in patients.

**Figure 12:** Analysis of the effect of SonoVue galactography in the diagnosis of nipple discharge (^*∗*^represents a statistically significant difference compared with conventional ultrasound, *P* < 0.05. ^*∗∗*^indicates that there is a significant difference compared with conventional ultrasound, *P* < 0.01).

## Data Availability

The simulation experiment data used to support the findings of this study are available from the corresponding author upon request.

## References

[1] Sun F., Liu Z., Zhang W. (2021). Clinical acupoint selection for the treatment of functional constipation by massage and acupuncture based on smart medical big data analysis. *Journal of Healthcare Engineering*.

[2] Cai Q., Mi Y., Chu Z., Zheng Y., Chen F., Liu Y. (2020). Demand analysis and management suggestion: sharing epidemiological data among medical institutions in megacities for epidemic prevention and control. *Journal of Shanghai Jiaotong University (Science)*.

[3] Agbehadji I. E., Awuzie B. O., Ngowi A. B., Millham R. C. (2020). Review of big data analytics, artificial intelligence and nature-inspired computing models towards accurate detection of COVID-19 pandemic cases and contact tracing. *International Journal of Environmental Research and Public Health*.

[4] Zhang Q. Phase-domain deep patient-ECG image learning for zero-effort smart health security.

[5] Wu Y., Zhang S., Dong Y. (2021). Therapeutic effect of electronic endoscopic hematoma removal on hypertensive basal ganglia cerebral hemorrhage based on smart medical technology. *Journal of Healthcare Engineering*.

[6] Peerapornratana S., Manrique-Caballero C. L., Gómez H., Kellum J. A. (2019). Acute kidney injury from sepsis: current concepts, epidemiology, pathophysiology, prevention and treatment. *Kidney International*.

[7] Kellum JA. (2019). Sepsis-associated acute kidney injury: a problem deserving of new solutions. *Nephron*.

[8] Li Y. (2021). Medical image fusion method by deep learning. *International Journal of Cognitive Computing in Engineering*.

[9] Liu D., Tang S., Gan L., Cui W. (2021). Renal-Protective effects and potential mechanisms of traditional Chinese medicine after ischemia-reperfusion injury. *Evidence Based Complementary Alternatative Medicine*.

[10] Li X., Yao L., Zeng X. (2021). miR-30c-5p alleviated pyroptosis during sepsis-induced acute kidney injury via targeting TXNIP. *Inflammation*.

[11] Zhuo Y. (2021). Tanshinone I exerts cardiovascular protective effects in vivo and in vitro through inhibiting necroptosis via Akt/Nrf2 signaling pathway. *Chinese Medicine*.

[12] Wu X., Sun W., Tan M. (2019). Noncoding RNAs in steroid-induced osteonecrosis of the femoral head. *BioMed Research International*.

[13] Zhang X. (2020). Administration of mircoRNA-135b-reinforced exosomes derived from MSCs ameliorates glucocorticoid-induced osteonecrosis of femoral head (ONFH) in rats. *Journal of Cellular and Molecular Medicine*.

[14] Zhou W., Qu “M. (2019). New advances in stem cell therapy for osteonecrosis of the femoral head. *Current Stem Cell Research & Therapy*.

[15] Li T. X. (2019). Prediction of collapse using patient-specific finite element analysis of osteonecrosis of the femoral head. *Journal of Orthopaedic Surgery*.

[16] Hatanaka H., Motomura G., Ikemura S. (2019). Differences in magnetic resonance findings between symptomatic and asymptomatic pre-collapse osteonecrosis of the femoral head. *European Journal of Radiology*.

[17] Zhu L. (2020). An automatic classification of the early osteonecrosis of femoral head with deep learning. *Current Medical Imaging*.

[18] Lv Z. H., Liang Q. (2020). Analysis of healthcare big data. *Future Generation Computer Systems*.

[19] Feng J. H. (2021). The anti-inflammatory and the antinociceptive effects of mixed agrimonia pilosa ledeb. And salvia miltiorrhiza bunge extract. *Plants (Basel)*.

[20] Chen L. (2021). Effects of tanshinone combined with valsartan on hypertensive nephropathy and its influence on renal function and vascular endothelial function. *American Journal of Translational Research*.

[21] Zhang Y., Lu P. (2021). Traditional Chinese medicine combined with pulmonary drug delivery system and idiopathic pulmonary fibrosis: rationale and therapeutic potential. *Biomedicine & Pharmacotherapy*.

[22] Luo P., Huang Y. (2021). Dihydrotanshinone I is effective against drug-resistant Helicobacter pylori in vitro and in vivo. *Antimicrob Agents Chemother*.

[23] Hua K. C. (2019). The efficacy and safety of core decompression for the treatment of femoral head necrosis: a systematic review and meta-analysis. *Journal of Orthopaedic Surgery and Research*.

[24] Wang Y., Ma J. X. (2019). Correlation between reduction quality of femoral neck fracture and femoral head necrosis based on biomechanics. *Journal of Orthopaedic Surgery and Research*.

[25] Li D., Li M. (2016). Core decompression or quadratus femoris muscle pedicle bone grafting for nontraumatic osteonecrosis of the femoral head: a randomized control study. *Orthopaedics*.

[26] Yoon J. Y., Lee S. J., Yoon K. S., Yoon P. W. (2020). The diagnostic value of SPECT/CT in predicting the occurrence of osteonecrosis following femoral neck fracture: a prospective cohort study. *BMC Musculoskeletal Disorders*.

[27] Huang Z. (2020). Dynamic evolution of osseous structure in osteonecrosis of the femoral head and dynamic collapse risks: a preliminary CT image study. *Journal of Orthopaedic Surgery and Research*.

[28] Hu M., Zhong Y. (2021). Fuzzy system based medical image processing for brain disease prediction. *Frontiers in Neuroscience*.

[29] Chen R. (2020). Combined predictive value of the risk factors influencing the short-term prognosis of sepsis. *Zhonghua Wei Zhong Bing Ji Jiu Yi Xue*.

